# Natural Antioxidants Improve the Vulnerability of Cardiomyocytes and Vascular Endothelial Cells under Stress Conditions: A Focus on Mitochondrial Quality Control

**DOI:** 10.1155/2021/6620677

**Published:** 2021-01-22

**Authors:** Xing Chang, Zhenyu Zhao, Wenjin Zhang, Dong Liu, Chunxia Ma, Tian Zhang, Qingyan Meng, Peizheng Yan, Longqiong Zou, Ming Zhang

**Affiliations:** ^1^Wangjing Hospital, China Academy of Chinese Medical Sciences, China; ^2^Guang'anmen Hospital, Chinese Academy of Traditional Chinese Medicine, Beijing, China; ^3^College of Pharmacy, Ningxia Medical University, Ningxia, China; ^4^China Academy of Chinese Medical Sciences, Institute of the History of Chinese Medicine and Medical Literature, Beijing, China; ^5^Shandong Analysis and Test Centre, Qilu University of Technology, Jinan, China; ^6^Shandong University of Traditional Chinese Medicine, Jinan, Shandong, China; ^7^Chongqing Sanxia Yunhai Pharmaceutical Co., Ltd., Chongqing, China

## Abstract

Cardiovascular disease has become one of the main causes of human death. In addition, many cardiovascular diseases are accompanied by a series of irreversible damages that lead to organ and vascular complications. In recent years, the potential therapeutic strategy of natural antioxidants in the treatment of cardiovascular diseases through mitochondrial quality control has received extensive attention. Mitochondria are the main site of energy metabolism in eukaryotic cells, including myocardial and vascular endothelial cells. Mitochondrial quality control processes ensure normal activities of mitochondria and cells by maintaining stable mitochondrial quantity and quality, thus protecting myocardial and endothelial cells against stress. Various stresses can affect mitochondrial morphology and function. Natural antioxidants extracted from plants and natural medicines are becoming increasingly common in the clinical treatment of diseases, especially in the treatment of cardiovascular diseases. Natural antioxidants can effectively protect myocardial and endothelial cells from stress-induced injury by regulating mitochondrial quality control, and their safety and effectiveness have been preliminarily verified. This review summarises the damage mechanisms of various stresses in cardiomyocytes and vascular endothelial cells and the mechanisms of natural antioxidants in improving the vulnerability of these cell types to stress by regulating mitochondrial quality control. This review is aimed at paving the way for novel treatments for cardiovascular diseases and the development of natural antioxidant drugs.

## 1. Introduction

Mitochondria are double-membrane-bound organelles that play an important role in the energy homeostasis of eukaryotic cells, including cardiomyocytes and endothelial cells [1]. According to the physiological needs in different living environments, mitochondria regulate their quantity and morphology [2]. With changes in the physiological environment, mitochondria can perform specific physiological processes related to quantity, morphology, and quality to maintain their structure and function. This process, termed “mitochondrial homeostasis,” is an important prerequisite for mitochondrial quality control (MQC) [3, 4].

Under oxidative stress, ischaemia, hypoxia, inflammation, and other stress conditions, mitochondrial homeostasis is disrupted [5]. This results in a disbalance of MQC, which affects mitochondrial quality and quantity, which can further lead to mitochondrial dysfunction and enhanced vulnerability, and induce apoptosis in cells [6, 7]. In the process of MQC, mitochondria can regulate their accumulation by decreasing enzyme activity and through mitochondrial fusion/fission and mitophagy to ensure normal physiological functionality [8, 9]. MQC plays an important role in maintaining the physiological functions of myocardial and endothelial cells and has attracted extensive attention in the treatment of cardiovascular diseases (CVDs) in recent years. MQC can be regulated by natural antioxidants in the treatment of CVDs and can further maintain the normal function of mitochondria.

Antioxidants are substances that prevent the harmful effects of oxygen. Antioxidants capture and neutralise free radicals to reduce damage to the body and organs. Antioxidants are made by the body but can also be supplied by plants or drugs. Natural antioxidants have long been used by humans [10]. They are found in many Chinese herbal and natural medicines and can effectively remove reactive oxygen species (ROS) and maintain the oxidation/antioxidation balance in cells and mitochondria. They can rapidly reach lesion sites and react with free radicals and have the characteristics of high safety, strong antioxidant capacity, and limited side effects [11]. Thus, natural antioxidants can significantly delay or inhibit ROS-induced oxidative damage. They can reduce excessive ROS production and improve the ability of cellular and mitochondrial antioxidant systems to scavenge free radicals, quench ^1^O_2_, and break down H_2_O_2_ [12]. They can regulate the redox state of cells and terminate oxidation processes by inhibiting the initiation and extension of redox reactions [13].

Recent studies have revealed that natural antioxidants can protect myocardial cells and endothelial cells via MQC under various stress conditions. In this review, the latest findings on the regulation of MQC based on *in vivo* and *in vitro* studies are discussed. In addition, the mechanisms of natural antioxidants of different types and sources in improving the vulnerability sensitivity of cardiomyocytes and endothelial cells under stress by regulating MQC are explored.

## 2. Method and Strategy

The literature on the advantages and mechanisms of natural antioxidants in improving cardiomyocyte and endothelial cell vulnerability through MQC published before November 2020 was searched in the Web of Science, MEDLINE, PubMed, Scopus, Google Scholar, and China National Knowledge Infrastructure databases. Keywords included “natural plants and mitochondrial quality control,” “natural antioxidants and oxidative stress,” “natural antioxidants and cardiomyocytes/endothelial cells,” “active ingredients of natural drugs and oxidative stress,” “natural plants,” and “cardiomyocytes/endothelial cells.” Original research articles related to natural antioxidants, MQC, and cardiomyocytes and endothelial cells were selected.

## 3. MQC

In 2019, a study published in *Nature* revealed that MQC defects can lead to CVDs and emphasised the importance of MQC [14]. MQC comprises mitochondrial autophagy, mitochondrial biosynthesis, mitochondrial fusion/fission, the mitochondrial respiratory chain, and the mitochondrial antioxidant system. MQC ensures the normal operation of the mitochondrial network and regulates timely mitochondrial turnover to maintain a stable quantity and quality of mitochondria in cardiomyocytes and endothelial cells [15]. Via MQC, mitochondria can regulate their numbers through mitochondrial fusion/fission, deliver damaged mitochondria or incorrectly folded proteins to lysosomes for degradation through mitophagy, and produce new mitochondria through biosynthesis. All MQC processes function independently as well as interact with each other to meet the energy demands of myocardial cells and endothelial cells under various conditions.

### 3.1. Regulatory Mechanism of MQC in Cardiomyocytes

Mitochondria comprise 25–30% of the myocardial cell volume and are widely distributed in the cell body and around the nucleus. The mammalian mitochondrial genome has 37 genes, 13 of which encode polypeptide subunits of enzyme complexes of the oxidative phosphorylation system, which provides more than 95% of the myocardial energy requirement for adenosine triphosphate (ATP) production [16, 17]. Mitochondria are the main organelles that mediate the energy production and apoptosis of cardiomyocytes [18, 19]. Because of the high energy requirement of myocardial cells, MQC is very important in these cells.

In a clinical study of 156 myocardial biopsy specimens, a single cardiomyocyte with obvious mitochondrial malformations was found in four samples [20]. The mitochondrial malformations in these four cardiomyocytes were accompanied by nuclear hypertrophy and/or sparse myofibrils. The malformations induced various disorders, including myocarditis, dilated cardiomyopathy, amyloidosis, and heart failure, all of which were accompanied by left ventricular systolic dysfunction [20].

Changes in mitochondrial quality and quantity directly affect the viability of cardiomyocytes and indirectly affect the pathological changes in myocardial diseases. As dynamic organelles, mitochondria can reshape their morphology under stress in myocardial infarction [21]. This reshaping of mitochondrial morphology (mitochondrion fission and fusion) is closely related to the expression of dynamin-related protein 1 (Drp-1) and mitofusin 1(Mfn1). Overexpression of Drp-1 and a decrease in Mfn1 expression in cardiomyocytes can destroy the mitochondrial fission/fusion balance and directly affect the contractility and function of cardiomyocytes [19]. Therefore, MQC plays an important role in myocardial cells.

### 3.2. Regulatory Mechanism of MQC in Endothelial Cells

In contrast to cardiomyocytes with their high energy demand, endothelial cells require less energy, and accordingly, their mitochondria account for only 2–6% of the cytoplasmic volume. The mitochondrial content of endothelial cells varies by the vascular bed and is higher in active endothelial cells. For example, endothelial cells at the blood-brain barrier are relatively active, and their mitochondrial content is as high as 8–11% [22].

The mitochondrial distribution in endothelial cells influences cell signal transduction. Under physiological conditions, mitochondria of endothelial cells are in a stable dynamic equilibrium state. Hypoxia-induced perinuclear aggregation of mitochondria can lead to the accumulation of mitochondrial (mt) ROS and induce transcription of the vascular endothelial growth factor gene [23]. Mitofusin-1 (Mfn1) is a mediator of mitochondrial fusion. When endothelial cells are injured by oxidative stress, the *Mfn1* mRNA expression is inhibited, resulting in the disbalance of mitochondrial fusion/fission in endothelial cells, reducing the quality of mitochondria and the function of endothelial cells [24, 25].

Peroxisome proliferator-activated receptor-gamma coactivator 1 alpha (PGC-1*α*) is abundant in endothelial cells and participates in the formation of mitochondria. In addition, it plays roles in antiapoptosis and anti-inflammation, improving the bioavailability of nitric oxide in endothelial cells. PGC-1*α* can increase the expression of uncoupling protein 2 and mitochondrial antioxidant enzymes, which is crucial for MQC and repair of oxidative damage in endothelial cells [26, 27].

Numerous studies have revealed that natural antioxidants can protect myocardial cells and endothelial cells under stress through the regulation of MQC. MQC is involved in cell protection against oxidative stress, inflammation, ischaemia/reperfusion (I/R), hypoxia/reoxygenation (H/R), high glucose, and lipid toxicity, and improves the vulnerability of myocardial cells and endothelial cells under stress.

## 4. Oxidative Stress

Oxidative stress is a state of imbalance between oxidation and antioxidation *in vivo* mediated by ROS [28]. Oxidative stress is considered an important cause of human ageing and various diseases and is a major factor leading to the apoptosis and death of myocardial cells and vascular endothelial cells [29]. Under oxidative stress, the efficiency of mitochondrial ATP synthesis strongly decreases and while ROS excessively accumulate, leading to the destruction of the interaction between mitochondria and the endoplasmic reticulum, thus accelerating apoptosis [30]. MQC can regulate the contractility, necrosis, and apoptosis of cardiomyocytes and endothelial cells under oxidative stress.

### 4.1. Effect of mtROS on MQC

Mitochondria are the main oxygen- (O_2_-) consuming sites in cells and the main source of ROS [31]. The mitochondrial respiratory chain, also known as the electron transport chain, is the core of mitochondrial energy production. Electron transport between respiratory chain complexes is coupled to proton transport through the mitochondrial membrane, resulting in the electrochemical gradient required for ATP synthesis [32, 33]. In addition, the respiratory chain is the main source of mitochondrial ROS production. ROS are a by-product of electron transfer in the respiratory chain. They are mainly produced by NADH: ubiquinone oxidoreductase and cytochrome C (cytC) oxidoreductase in the respiratory chain [34].

While mitochondria are the main source of ROS production, they are also the primary target of ROS attack. Proinflammatory factors released in response to excessive ROS production can directly damage mitochondrial respiratory chain function, reduce mitochondrial energy metabolism, and damage the mitochondrial antioxidant system, leading to further aggravation of oxidative stress damage [35, 36]. Excessive ROS production can also cause an abnormal opening of the mitochondrial membrane permeability transition pore (mPTP), which leads to an imbalance in mitochondrial membrane permeability transition and ion concentrations inside and outside the mitochondria. In addition, ROS activate various factors, including cytC, Bax, and caspase, to induce apoptosis of cardiomyocytes and endothelial cells [31, 37]. ROS-mediated oxidative stress can change mitochondrial structure and function, leading to excessive mitochondrial fission [38]. The qualitative and morphological damage of mitochondria caused by the imbalance of mitochondrial dynamics leads to apoptosis induction [39].

Endothelial cells isolated from a hypoxia-induced pulmonary hypertension rat model (such as microvascular endothelial cells) reportedly show excessive mtROS production, an imbalance in intracellular calcium (Ca^2+^) levels, and an increase in abnormal mitochondrial fission [40]. Inhibition of mtROS suppresses abnormal mitochondrial division in endothelial cells, whereas mtROS production is induced in microvascular endothelial cells of normoxic rats, which increases the level of abnormal mitochondria [40]. It has been suggested that oxidative stress-mediated by mtROS may lead to an imbalance in mitochondrial Ca^2+^, division, and respiratory function. Natural antioxidants, which can scavenge free radicals and inhibit excessive ROS production, highlight the advantages and potential of regulating MQC.

### 4.2. Role of the Mitochondrial Antioxidant System in MQC

Myocardial cells and endothelial cells are vulnerable to oxidative stress [41]. To suppress ROS-mediated oxidative stress and mitochondrial damage, mitochondria have a complete antioxidant system and an ROS-scavenging system [42]. The mitochondrial antioxidant system comprises superoxide dismutase (SOD), glutathione peroxidase (GSH-Px), and peroxiredoxin (PRX) [43]. They can directly scavenge free radicals or convert highly reactive superoxide radicals into hydrogen peroxide, which can be further eliminated by catalase and the GSH-Px and peroxiredoxin/thioredoxin systems [44].

SOD is the most important antioxidant in mitochondria and is located in the mitochondrial matrix. It reduces oxidative free radicals to H_2_O_2_, eliminates large amounts of O_2_^−^, and prevents superoxide-induced damage to mitochondrial (mt) DNA and proteins [45]. GSH is the most abundant nonprotein sulfhydryl and has a wide range of antioxidant effects. It mainly reduces lipid peroxides induced by ROS and hydroxyl groups [46] and reduces H_2_O_2_ to H_2_O [47]. Together, these antioxidants constitute the mitochondrial antioxidant system. As shown in Figure 1 and Table 1, H/R, I/R, lipid toxicity, inflammation, high glucose, and other stress conditions are accompanied by the massive release free radicals, such as H_2_O_2_, NO, OH, and ONOO^−^, which also leads to the excessive production of ROS and reactive nitrogen species (RNS). The excessive production of ROS and RNS further reduces the activity of antioxidant enzymes, including SOD, GSH, CAT, GSH-Px, and PRX. The mitochondrial antioxidant system cannot control ROS-mediated oxidative stress damage, leading to the appearance of oxidative stress markers, such as malondialdehyde (MDA), 8-hydroxyguanosine, and 8-2′-hydroxydeoxyguanosine. This may be the main pathological mechanism of cardiomyocyte and vascular endothelial cell damage caused by different stress conditions.

Natural antioxidants have become key candidate drugs for MQC regulation to repair mitochondrial oxidative damage and improve the vulnerability of cardiomyocytes and endothelial cells after the destruction of the mitochondrial antioxidant system.

### 4.3. Natural Antioxidants That Protect Myocardial and Endothelial Cells through MQC under Oxidative Stress Conditions

#### 4.3.1. *Panax notoginseng* Saponins

*P. notoginseng* saponins are active components in *P. notoginseng*, which is used as a natural medicinal herb, with strong antioxidant effects [48]. *P. notoginseng* saponins significantly reverse the downregulation of forkhead box O3a and Mn-SOD, upregulate PGC-1*α*, LC3-II, and Beclin-1, regulate PGC-1*α* expression and mitophagy, reduce ROS-mediated oxidative damage, improve mitochondrial dysfunction caused by ageing and morphological changes in rat myocardium, and inhibit the apoptosis of cardiomyocytes [49].

#### 4.3.2. Astragaloside IV

Astragaloside IV (AS-IV) is a natural antioxidant found in rhizomes of *Astragalus membranaceus*. It has various pharmacological activities, including antioxidation, anti-inflammation, and antitumour activities [50]. AS-IV significantly inhibits doxorubicin-induced ROS overproduction and release of lactate dehydrogenase (LDH), creatine kinase MB isoenzyme, and cytC, increases the activities of succinate dehydrogenase and ATP synthase, and restores ATP synthesis [51]. Further, AS-IV significantly inhibits mitochondrial apoptosis pathway activation by inducing phosphorylation of phosphatidylinositol 3-kinase (PI3K)/Akt, and the PI3K inhibitor LY294002 significantly inhibits the antiapoptotic effect of AS-IV. [51].

#### 4.3.3. Cabbage Extract

Extract of *Brassica oleracea* L., a member of the cabbage family (Brassicaceae), has various pharmacological effects, and its antioxidant effect is exploited in the treatment of various CVDs [52]. Recent *in vitro* research has revealed that cabbage extract inhibits ROS production and increases SOD-1, catalase (CAT), and GPX activities. It inhibits the overactivation of MAPK proteins (ERK1/2, JNK, and P-38) and apoptosis of H9C2 cardiomyocytes without any cytotoxicity [53]. This suggests that cabbage extract can regulate MQC to reduce H_2_O_2_-induced oxidative stress injury in H9C2 cardiomyocytes and can be used in dietary replacement therapy to protect cardiomyocytes.

#### 4.3.4. Homoeriodictyol

Homoeriodictyol is an effective active component of mistletoe that has many pharmacological effects, including improvement of microcirculation, antioxidation, and antiplatelet aggregation [54, 55]. Nuclear factor erythroid 2-related factor 2 (Nrf2) plays an important role in cytoprotection from ROS-induced oxidative damage. An *in vitro* study found that homoeriodictyol can upregulate the expression of Nrf2. It further corrects mitochondrial membrane potential (MMP) loss, inhibits the release of cytC and apoptosis-inducing factor, inhibits the overexpression of caspase-3/9 induced by H_2_O_2_, increases the expression of Bcl-2 and Bcl-xL, and suppresses apoptosis of endothelial cells under oxidative stress [56].

#### 4.3.5. Tanshinone IIA

Tanshinone IIA is a lipid-soluble phenanthrenequinone compound in *Salvia miltiorrhiza* that has antibacterial, anti-inflammatory, antioxidant, and other pharmacological effects [57]. Tanshinone IIA protects bovine retinal endothelial cells from oxidative stress induced by methylglyoxal [22]. In endothelial cells, it significantly reduces abnormal mitochondria, increases the mRNA expression of *Mfn1* and *OPA1*, inhibits mitochondrial fusion, repairs oxidative stress injury, and increases cellular activity. siRNA-mediated silencing of *GLO1* inhibits the induction of mitochondrial fusion by tanshinone IIA. Thus, it was concluded that tanshinone IIA treatment regulates MQC by increasing the level of GLO1 and improves the vulnerability of endothelial cells under oxidative stress [22, 58].

#### 4.3.6. Ligustrazine

Ligustrazine is an alkaloid in *Ligusticum chuanxiong*, Hort. It has strong antioxidant, antiplatelet aggregation, and microcirculation improvement effects [59]. Ligustrazine improves oxidative stress injury induced by high homocysteine, restores the MMP, inhibits the release of cytC from the mitochondria into the cytoplasm, reduces the level of LDH, inhibits apoptosis, and improves the cellular activity in human umbilical vein endothelial cells (HUVECs) [60].

#### 4.3.7. Resveratrol

Resveratrol is a polyphenol compound abundant in peanut, *Polygonum cuspidatum*, and mulberry. It has strong antioxidant activity and is commonly used in the treatment of CVDs [61, 62]. Resveratrol protects against oxidative damage of MQC in endothelial cells. It activates TyrRS-PARP1 signalling and increases the expression of Mfn1, Mfn2, and OPA1. Moreover, it inhibits excessive mitochondrial fission, restores the MMP, and inhibits apoptosis in HUVECs. The regulatory effect of resveratrol on mitochondrial fission/fusion and its protective effect on endothelial cells were affected by siRNA interference of *TyrRS* and *PARP1*, indicating that resveratrol regulates mitochondrial fission/fusion through TyrRS-PARP1 signalling [63].

Resveratrol increases the enzyme activities of isocitrate dehydrogenase 2 (IDH2), GSH-Px, and manganese SOD (SOD2) via SIRT3 signalling, and upregulates the expression of *Atp6*, *CO1*, *ND2*, and *ND5* mediated by forkhead box O3a. It inhibits ROS production in mitochondria, enhances the activities of electron chain complex I and ATP synthesis, restores the MMP, and inhibits apoptosis in HUVECs. In addition, it enhances the phosphorylation of adenosine monophosphate-activated protein kinase (p-AMPK) and the expression of PGC-1*α* and SIRT3. MQC regulation and the protective effect of resveratrol on endothelial cells were inhibited by treatment with an AMPK inhibitor or siRNAs against *AMPK*, *PGC-1α*, and *SIRT3*. This suggests that resveratrol can reduce the oxidative damage of endothelial cells by regulating MQC, which may be mediated by the AMPK-PGC-1*α*-SIRT3 pathway [64].

#### 4.3.8. Luteolin

Luteolin is a flavonoid compound widely found in pepper, chrysanthemum, and other plants, and has a strong antioxidant effect [65]. Luteolin protects endothelial cells from oxidative stress injury induced by H_2_O_2_ by regulating ROS-mediated p38MAPK/NF-*κ*B and Ca^2+^-induced mitochondrial apoptosis signalling. It strongly suppresses increases in intracellular Ca^2+^, restores the MMP, regulates p53 phosphorylation and the Bcl-2/Bax ratio, and inhibits cytC release, caspase-3 overexpression, and apoptosis in endothelial cells [66].

#### 4.3.9. Grape Seed Proanthocyanidins

Grape seed proanthocyanidins are extracted from the seeds of grapes (*Vitis vinifera*). As natural polyphenol compounds and natural antioxidants, grape seed proanthocyanidins scavenge free radicals and have antioxidant and anti-inflammatory effects [67, 68]. Grape seed proanthocyanidins inhibit excessive ROS production, restore the MMP, improve the respiratory function of mitochondria, reduce the level of 8-hydroxydeoxyguanosine (8-OHdG), enhance endothelial nitric oxide synthase (eNOS) and VE-cadherin expression, and inhibit apoptosis in endothelial cells. In HUVECs, they improve oxidative stress injury induced by indole sulphate [69].

## 5. Hypoxia

Hypoxia is a pathological process comprising abnormal changes in tissue metabolism, function, and morphology due to insufficient O_2_ supply or respiratory dysfunction [70]. Hypoxia is a common mechanism in the development of various diseases. Hypoxia in the brain and heart is also the primary cause of death. O_2_ plays an important role in the regulation of metabolism, energy production, and internal homeostasis [71]. If tissues, organs, and cells cannot adapt to the lack of O_2_ supply, excessive ROS production and oxidative stress damage may occur under hypoxia, which leads to MQC imbalance, cell apoptosis, and tissue necrosis [72].

### 5.1. Effects of Hypoxia on ROS

Mitochondria are very sensitive to the O_2_ concentration in the living environment. The balance between O_2_ supply and consumption in the body is the physiological basis for maintaining normal mitochondrial respiratory chain function. In mitochondria, long-term insufficient O_2_ supply will directly affect O_2_ exchange, transport, and release in tissues, resulting in intracellular hypoxia [73].

Under hypoxia, there is insufficient O_2_ to serve as an electron acceptor in oxidative phosphorylation, and thus, free electrons increase and excessive ROS are generated. ROS accumulation can lead to oxidative damage of macromolecules and abnormal mPTP opening [74]. Oxidative phosphorylation dysfunction under hypoxia can also lead to mitochondrial respiratory chain damage [75, 76]. Excessive mtROS production due to respiratory chain injury can induce cell signal transduction pathways and cause lipid peroxidation of the cell membrane, resulting in apoptosis and homeostasis imbalance [77]. Myocardial myofibrillar protein oxidation by ROS suppresses cardiac systolic and diastolic function, resulting in the decline of cardiac function [78, 79].

### 5.2. Effect of Hypoxia on MQC

Hypoxia affects not only mitochondrial respiratory chain function but also the morphology and quality of mitochondria, and induces functional and morphological changes in the peripheral mitochondria. It also causes damage to lipids, proteins, and DNA, resulting in MMP loss, cytC release, and caspase-3/9 activation, thus increasing the vulnerability of cardiomyocytes and endothelial cells [80].

ROS directly affect mitochondrial Ca^2+^ homeostasis, lead to dysfunction of the mitochondrial Ca^2+^ uniporter, and induce mitochondrial Ca^2+^ overload [81]. Mitochondrial Ca^2+^ transport, mPTP opening, and caspase-3/7/8/9 activity were significantly decreased after siRNA treatment. The imbalance of MQC caused by H/R is mainly related to the dysregulation of the mitochondrial Ca^2+^ uniporter [82].

MQC is determined by mitochondrial fission/fusion balance, mitophagy, mitochondrial respiratory function, and mitochondrial biosynthesis. These processes are enhanced by OPA1 knockout and attenuated by OPA1 overexpression [83]. The antiapoptotic effect of hypoxic postconditioning cannot be attenuated only by SOD and CAT in the mitochondrial antioxidant system [83]. Therefore, it is necessary to find natural antioxidants that can regulate MQC to improve cell vulnerability under hypoxia.

### 5.3. Natural Antioxidants That Protect Myocardial and Endothelial Cells through MQC under Hypoxia

#### 5.3.1. Ginseng Polysaccharide

Ginseng polysaccharide is an acidic polysaccharide present in *Panax ginseng*. As a natural antioxidant, ginseng polysaccharide has good anti-inflammatory, antitumour, and antithrombotic effects [84, 85]. It is effective in protecting myocardial cells from H/R injury. It restores mitochondrial energy metabolism and the MMP, blocks mitochondrial cytC release, increases ATP production, and regulates the O_2_ consumption rate. It also induces glucocorticoid receptor and oestrogen receptor expression activates the reperfusion injury salvage kinase (RISK) pathway, increases the production of nitric oxide by increasing eNOS and iNOS expression, and protects endothelial cells [85].

#### 5.3.2. Isoquercetin

Isoquercetin is a flavonoid isolated from the seed pod of *Cercis canadensis* and exists in plants such as *Eucommia ulmoides* Oliv. and mulberry leaf. The pharmacological activities of many plants are related to isoquercetin [86, 87]. Isoquercetin has a strong antioxidant effect through which it inhibits ROS production in mitochondria, improves energy metabolism in mitochondria, inhibits cytC release and apoptosis, and protects myocardial cells from damage induced by hypoxia-induced oxidative stress [88].

#### 5.3.3. *Bauhinia championii* Flavone

*Bauhinia championii* flavone scavenges free radicals and has an antiarrhythmic effect [89, 90]. It improves mitochondrial dysfunction, alleviates H9C2 cardiomyocyte apoptosis induced by H/R, significantly inhibits ROS production, increases ATP synthesis, and inhibits abnormal mPTP opening. In addition, it inhibits the mitochondrial translocation of Bax, cytC release, and caspase-3 expression, increases PI3K and Akt phosphorylation, regulates the Bcl-2/Bax ratio, and inhibits H/R-induced apoptosis in cardiomyocytes. LY294002, a specific inhibitor of PI3K, partially reversed the regulatory effects of *B. championii* flavone on cardiomyocytes and MQC, suggesting that the flavone improves mitochondrial function through PI3K/Akt signalling, thus reducing H/R-induced cardiomyocyte apoptosis [91].

#### 5.3.4. Schisandrin/Schisandrin B

Schisandrin and schisandrin B are active lignoid substances extracted from *Schisandra chinensis*. They have anti-inflammatory, antioxidation, antitumour, and immune-regulatory effects [92, 93]. Both schisandrin and schisandrin B protect H9C2 cardiomyocytes from apoptosis induced by H/R by inhibiting abnormal mPTP opening and cytC release, increasing the cleavage of caspase-3 and poly ADP ribose polymerase, and enhancing GSH expression [94].

#### 5.3.5. Picroside

Picroside is an active component in *Picrorhiza* sp. that has strong anti-inflammatory and antioxidant effects [95, 96]. Picroside significantly inhibits ROS production in mitochondria, inhibits mPTP opening, increases the MMP, inhibits cytC release from the mitochondria downregulates caspase-3, and suppresses cardiomyocyte apoptosis induced by H/R in cardiomyocytes, suggesting that picroside improves cardiomyocyte activity by reducing ROS production [97].

#### 5.3.6. Anthocyanins

Anthocyanins are water-soluble pigments that are widely present in plant vacuoles and belong to the flavonoid compounds. They are derived from chlorophyll and have anti-inflammatory, antioxidant, and antiallergic effects [98, 99]. As natural antioxidants, anthocyanins improve oxidative stress injury induced by peroxynitrite, restore the MMP, inhibit caspase-3/9 expression and Bax transport to the nucleus, and improve the function of endothelial cells [100].

## 6. Ischaemia/Reperfusion

Ischaemia-induced myocardial, vascular, or other organ tissue damage is the main cause of cardiovascular and cerebrovascular diseases, such as coronary atherosclerosis, myocardial infarction, and stroke [101]. In the process of I/R, the main factor of tissue damage is not ischaemia itself, but the ROS-induced oxidative stress damage in cells (such as myocardial cells and vascular endothelial cells) after the recovery of blood supply, leading to tissue damage or necrosis [102]. During I/R, ROS-induced mitochondrial Ca^2+^ imbalance, mitochondrial respiratory chain dysfunction, and energy metabolism disorders are the main causes of increased vulnerability of myocardial cells and endothelial cells [103].

### 6.1. Effect of I/R on mtROS

As highly dynamic organelles, mitochondria constantly undergo fusion and fission, and the balance between these processes plays an important role in cell homeostasis [104]. The fusion and fission of mitochondria are mediated by fusion and cleavage proteins. During I/R, ROS-mediated oxidative stress leads to imbalances in mitochondrial fusion/mitogen protein expression and posttranslational modification regulation, resulting in abnormal mitochondrial fusion/fission and MQC imbalance [105].

When mitochondrial dysfunction occurs, the defence mechanism of the mitochondrial antioxidant system is also affected. ROS production exceeds the scavenging capacity of the mitochondrial antioxidant system, which results in oxidative stress damage [106]. The explosive increase in ROS may be caused by respiratory chain decoupling. I/R induces the activities of nicotinamide adenine dinucleotide phosphate oxidase (NOX), xanthine oxidase, and NOS, enhancing ROS production [107]. Excessive ROS trigger cell apoptosis and aggravate tissue damage by inducing mPTP opening, activating various enzymes and transcription factors, and stimulating inflammatory reactions and mtDNA damage [108]. Therefore, the imbalance of MQC caused by ROS plays an important role in the tissue damage caused by I/R.

### 6.2. Effects of I/R on MQC

I/R affects MQC in various ways. In the ischaemic state, aerobic oxidation is inhibited, which leads to a serious shortage of ATP synthesis. Consequently, energy metabolism in the heart is dominated by anaerobic glycolysis [109]. Anaerobic glycolysis produces a large amount of lactic acid, resulting in a decrease in Na^+^/K^+^-ATPase activity and an increase in intracellular Na^+^. The Na^+^/Ca^2+^ pump is then activated and the Ca^2+^ concentration in the cytoplasm increases rapidly. To maintain intracellular Ca^2+^ homeostasis, mitochondria import excess Ca^2+^ from the cytoplasm, which results in an overload of mitochondrial Ca^2+^ and changes in membrane permeability, leading to mitochondrial swelling and irreversible damage [110, 111]. A high concentration of Ca^2+^ also enhances the ATP hydrolysis activity of F0F1 ATPase and inhibits the synthesis of mitochondrial ATP through Ca^2+^ binding to ATPase inhibitor protein [112].

Under the condition of reperfusion, cells reabsorb O_2_ from the blood, which leads to explosive ROS formation and serious protein and lipid peroxidation, resulting in a decline in mitochondrial cytC oxidase and ATP synthase activities, thus affecting respiratory chain function [113]. ROS also activate phospholipase, degrade membrane phospholipids, and damage the mitochondrial structure and respiratory chain function [114]. In conclusion, early correction of MQC imbalance and inhibition of ROS-mediated oxidative stress injury are important ways to improve the vulnerability of myocardial cells and endothelial cells under I/R.

### 6.3. Natural Antioxidants That Protect Myocardial and Endothelial Cells through MQC during I/R

#### 6.3.1. *Panax quinquefolium* Saponin

Abnormal mPTP opening is an important mechanism of myocardial injury induced by I/R [114]. *P. quinquefolium* saponin is the most abundant compound in *P. quinquefolium*. It reduces blood lipids, blood pressure, and lipid peroxidation, and is an effective natural antioxidant [115]. *P. quinquefolium* saponin improves the vulnerability of cardiomyocytes in the I/R state by regulating MQC. It effectively inhibits mPTP opening, regulates MMP depolarisation, increases the Bcl-2/Bax ratio, inhibits the translocation of mitochondrial cytC to the cytoplasm, protects mitochondrial structure, inhibits ROS production and caspase-9/3 expression, and suppresses apoptosis in cardiomyocytes under I/R injury [116].

#### 6.3.2. Ginsenoside Rg5

Ginsenoside Rg5 is a sterol present in ginseng with antioxidant activity [117]. Rg5 inhibits fatty acid oxidation, improves pyruvate dehydrogenase activity, and prevents cell acidification. Rg5 activates Akt signalling to regulate Drp-1, promotes mitochondrial hexokinase- (HK-) II binding, increases the permeability of cardiomyocytes to ATP/5, improves mitochondrial respiratory function and hypoxia tolerance, and improves the vulnerability of myocardial cells to ischaemia [118].

#### 6.3.3. Lycopene

Lycopene is an antioxidant that exists mainly in mature fruits of tomato (*Solanum lycopersicum*). It is one of the strongest natural antioxidants found in plants. Lycopene is far more effective in scavenging free radicals than other carotenoids and vitamin E [119, 120]. I/R injury increases the 8-OHdG content in cardiomyocytes, decreases mtDNA transcription, and results in mitochondrial energy metabolism disorder. Lycopene suppresses mtROS production, restores the protein expression of a key activator of mtDNA transcription (TFAM), and inhibits 8-OHdG expression, thus protecting cardiomyocytes from oxidative stress induced by I/R [121].

#### 6.3.4. *Cynomorium songaricum* Extract

*C. songaricum* Rupr. is a perennial fleshy parasitic herb. It contains flavonoids, triterpenoids, tannins, steroids, and organic acids. *C. songaricum* extract has free radical-scavenging, antihypoxia, and immunoregulatory effects [122, 123]. *In vivo* and *in vitro* studies have shown that *C. songaricum* extract protects H9C2 cells and rat myocardium by enhancing mitochondrial ATP production and the glutathione redox cycle, regulating MQC, and inhibiting LDH and caspase-3 expression [124].

#### 6.3.5. Quercetin

Quercetin is an antioxidant that exists in Berberidaceae and *Hypericum andraeanum* and has anti-inflammatory and immunomodulatory effects. It reduces blood pressure and improves capillary elasticity [125, 126]. Ang-II decreases the activity of HUVECs in a concentration-dependent manner. Quercetin inhibits Ang-II-induced damage to HUVECs in a concentration- and time-dependent manner. Quercetin restores the MMP, inhibits the translocation of cytC, and upregulates Bax and Bcl-2 and inhibits caspase-3/9 activation, thus inhibiting apoptosis in HUVECs [127].

## 7. High Glucose

With the increase in energy consumption per capita, lipid metabolism disorders caused by high glucose and CVD caused by oxidative stress are on the rise and have been widely studied [128]. These disorders are mainly due to MQC imbalance caused by hyperglycaemia and cardiomyocyte and vascular endothelial cell dysfunctions, including oxidative stress, increased glycation end products, coagulation, and fibrinolysis system dysfunction, which cause the accumulation of vascular substances, vascular stenosis, and atherosclerosis [129, 130]. Therefore, CVDs associated with diabetes mellitus are a major cause of death, which is closely related to high glucose-mediated MQC imbalance and cell dysfunction [131].

### 7.1. High Glucose- and ROS-Mediated Oxidative Stress

High glucose-induced vascular injury involves the polyol pathway, changes in redox status, an increase in diacylglycerol formation, and the accumulation of nonenzymatic glycation end products [132]. High glucose levels regulate multiple signalling pathways to induce apoptosis in cardiomyocytes and endothelial cells, mainly via ROS-mediated oxidative stress [133].

When blood glucose levels rise, insulin secretion from *β* cells in the pancreatic islets into the blood increases. Under normal physiological conditions, the surrounding tissues respond to insulin by increasing the expression of glucose transporters on the plasma membrane. However, consistent high glucose levels and consequent long-term high insulin levels will lead to insulin resistance [134]. High levels of insulin interfere with NOX4 signal transduction and enhance ROS production [135]. Thus, insulin resistance induced by high glucose indirectly leads to excessive ROS production and oxidative stress damage, which may be why high glucose levels can lead to type 2 diabetes mellitus complicated by CVD.

### 7.2. Effects of High Glucose on MQC in Cardiomyocytes and Endothelial Cells

Enhanced ROS in response to high glucose interferes with the mitochondrial electron transport chain, which increases the oxidation of coenzyme Q, thus forming peroxides. These peroxides react with nitrous oxide to form peroxynitrite (ONOO^−^), which leads to mitochondrial protein dysfunction, lipid oxidation, and DNA modification, eventually leading to cell apoptosis [136].

As the centre of glucose metabolism, mitochondria are likely to be affected by diabetes-related metabolic damage. Although the reasons for the increased risk of heart failure are multifactorial, high glucose-induced mitochondrial dysfunction in cardiomyocytes and endothelial cells plays a key role [137, 138]. Mitochondrial energy metabolism and dynamics defects, oxidative stress, Ca^2+^ homeostasis, and mitochondrion-induced cell death have been observed in diabetic myocardial mitochondria. Mitochondrial dysfunction seems to be the main cause of arrhythmia in diabetes mellitus [139].

In HUVECs treated with high glucose, the expression of Tom22 and OXPHOS was impaired and mitochondrial fusion was decreased, and deletion of Tom22 resulted in a decrease in mitochondrial fusion and ATP production and an increase in apoptosis in HUVECs [24]. Rotenone, an inhibitor of mitochondrial electron transport, suppresses excess ROS production in streptozotocin-induced diabetic rats that exhibited mitochondrial damage, loss of MMP, as well as increased caspase-3/9 activities and apoptosis [140]. High glucose levels induce apoptosis and MMP loss in HUVECs by enhancing Bax expression and suppressing Bcl-2 expression. Cells exposed to high levels of sugar release cytC in excess [141]. Therefore, regulation of the MQC imbalance induced by high glucose is a key target to improve the vulnerability of cardiomyocytes and endothelial cells in a high-glucose environment.

### 7.3. Natural Antioxidants That Protect Myocardial and Endothelial Cells through MQC under High-Glucose Conditions

#### 7.3.1. Naringin

Naringin is a dihydroflavonoid extracted from the dried outer peel of *Citrus grandis* (L.) Osbeck and *Citrus paradisi* Macfad. [142]. It has anti-inflammatory, antiviral, and antithrombotic effects [143]. Naringin significantly inhibits p38 and p53 phosphorylation induced by high glucose, restores the MMP, regulates Bax and Bak expression, prevents mitochondrial cytC release, increases Bcl-2 expression, and inhibits caspase-3/8/9 activation and apoptosis in H9C2 cells [144].

#### 7.3.2. Berberine

Berberine is a quaternary ammonium alkaloid in *Coptis chinensis*. It has various pharmacological activities, including antioxidative, hypoglycaemic, blood lipid-regulatory, blood pressure-lowering, and antiarrhythmia effects [145, 146]. Cardiomyocyte hypertrophy induced by type 2 diabetes mellitus is closely related to mitochondrial dysfunction. Berberine significantly improves mitochondrial fusion/fission imbalance and mitochondrial energy metabolism in H9C2 cells. It increases the level of mitophagy induced by high glucose levels by activating AMPK signalling, and promotes mitochondrial biosynthesis in H9C2 cells and improves the vulnerability of cardiomyocytes to high glucose [147].

#### 7.3.3. Cinnamaldehyde

Cinnamaldehyde is an organic aldehyde found in *Cinnamomum cassia*. It has antioxidant, vasodilatory, and blood pressure-lowering effects [148]. Transient receptor potential cation channel subfamily A member 1 (TRPA1) has an antioxidant effect. Cinnamaldehyde significantly reduces high glucose-induced ROS production, upregulation of nitrotyrosine, P22, and P47, and apoptosis in H9C2 cardiomyocytes. It upregulates Nrf2 and its target genes, heme oxygenase-1 (*HO-1*), *GPX-1*, and quinone oxidoreductase-1 (*NQO-1*). Hc030031, a TRPA1 inhibitor, abolishes the protective effect of cinnamaldehyde on cardiomyocytes. Cinnamaldehyde significantly reduces the levels of nitrotyrosine, fibrosis, and cardiomyocyte hypertrophy in rats and increased the expression of HO-1, GPX-1, NQO-1, and CAT in the myocardium of diabetic mice. Thus, it seems to protect cardiomyocytes against oxidative stress injury induced by high glucose through the TRPA1/Nrf2 pathway [149].

#### 7.3.4. Rosmarinic Acid

Rosmarinic acid is a water-soluble natural phenolic acid isolated from rosemary (*Rosmarinus officinalis*). It mainly exists in Labiatae, Arnebiaceae, and Cucurbitaceae. It is a natural antioxidant [150, 151]. Rosmarinic acid inhibits ROS production and abnormal mPTP activation induced by high glucose, as well as cytC release and caspase-3 activation. It protects H9C2 cells against apoptosis induced by high glucose. It increases STAT3 phosphorylation. siRNA-mediated knockdown of STAT3 inhibits the protective effect of rosmarinic acid on high glucose-induced apoptosis, indicating that rosmarinic acid improves mitochondrial function and inhibits cardiomyocyte apoptosis induced by high glucose through the STAT3 pathway [152].

#### 7.3.5. Resveratrol

Resveratrol inhibits high glucose-induced mtROS production in human coronary artery endothelial cells via the intracellular target protein deacetylase silent information regulator (SIRT)2/SIRT1 [153]. In endothelial cells, SIRT1 overexpression attenuates mtROS production and overexpression of RSV and SIRT1 significantly reduces the level of H_2_O_2_ and increased Mn-SOD and GSH expression in a concentration-dependent manner. Thus, resveratrol reduces mtROS production by activating SIRT1 and restoring the antioxidant defence mechanism of mitochondria, which implies the potential of new therapeutic methods targeting endothelial mitochondria in metabolic diseases [154].

#### 7.3.6. *Pleurotus nebrodensis* Extract

The fungus *P. nebrodensis* contains polysaccharides, vitamins, and other physiologically active substances that can regulate the physiological balance and enhance immune function in the human body [155]. *P. nebrodensis* extract improves high glucose-induced mitochondrial dysfunction in EA.hy926 endothelial cells. It inhibits the increase in electron transport chain complex I activity and decrease in ROS production induced by hyperglycaemia. It suppresses the oxidative damage of lipids and proteins, regulates imbalanced SOD and CAT activities, reduces the level of nitric oxide, restores mitochondrial function, and improves the vulnerability of endothelial cells to hyperglycaemia [153].

#### 7.3.7. Obtusin

Obtusin is an anthraquinone compound with antioxidant activity extracted from *Cassia obtusifolia* [156]. Obtusin inhibits high glucose-induced mitochondrial apoptosis in HUVECs and high glucose-induced ROS production. It decreases the MDA content and restores the activities of mitochondrial complexes I/III, CAT, and SOD. Obtusin restores the MMP and prevents the release of Omi/HtrA2 into the cytoplasm, thus protecting endothelial cells from apoptosis [157].

#### 7.3.8. Polydatin

Polydatin is a small-molecule compound in *Polygonum cuspidatum*, which is used as a medicinal herb. It has many biological functions, including antioxidation, anti-inflammation, and renal protection [158]. Methylglyoxal, an active metabolite of glucose, induces apoptosis of vascular cells in diabetic complications. Polydatin significantly inhibits ROS production induced by methylglyoxal, restores the MMP and mitochondrial morphological changes, and increases Akt phosphorylation, and it inhibits methylglyoxal-induced apoptosis of HUVECs. Polydatin improves the vulnerability of methylglyoxal-induced HUVECs at least in part by inhibiting oxidative stress, maintaining the mitochondrial function, and activating Akt signalling [159].

## 8. Inflammation

Inflammation is a defence response of tissues, including blood vessels, to injury and a physiological homeostatic response [160]. Normal inflammation can eliminate invasive organisms and foreign stimuli; however, excessive inflammation can damage cardiomyocytes and endothelial cells, leading to the occurrence of CVDs, such as myocarditis, atherosclerosis, acute myocardial infarction, vasculitis, and heart failure [161]. Different types of inflammatory reactions are involved in the development of CVDs. These inflammatory reactions are often related to ROS-mediated oxidative stress. Moreover, with the onset and development of inflammation, activated infiltrating immune cells and inflammatory resident cells will gradually increase the demand for mitochondrial energy, which will lead to hypoxia, mitochondrial energy metabolism dysfunction, and ROS production [162]. Furthermore, MQC imbalance and increased ROS levels lead to serious oxidative damage and promote the onset of inflammation.

### 8.1. Effect of Inflammation on ROS

As important intracellular messengers, ROS can activate various inflammatory signal transduction pathways. Oxidative stress can lead to MQC imbalance through direct cytotoxicity and promote the onset and development of local inflammatory responses [163]. Oxidative stress and inflammation are interdependent, especially in mitochondria. Excessive ROS production at inflammatory sites can lead to oxidative stress damage to mitochondria. Oxidative stress products can enhance inflammatory factor responses, and there are interactions between them. Mitochondria may be the “Trojan horse” of inflammation while maintaining the basic cellular functions [164].

Abnormal mitochondrial fission in endothelial cells can also lead to inflammation and oxidative stress. Inflammation may be inhibited via the regulation of the mitochondrial fission/fusion balance. In normal physiology, Drp-1 plays a beneficial role in maintaining the fission/fusion balance in endothelial cells. However, under inflammation, Drp-1 increases, resulting in excessive mitochondrial fission, which leads to chronic inflammation. When mitochondria are damaged by stress or bacterial toxins, NLRP3 is also activated, leading to an inflammatory state [165, 166]. Zhong et al. found that damaged mitochondria activate NLRP3 and NLRP3 activation which was inhibited when mitochondrial autophagy cleared abnormal mitochondria and damaged proteins [167]. mtROS can also induce NLRP3 activation. The oxidative effect of ROS on mtDNA during NLRP3 activation leads to a partial inflammatory potential of free, circulating mtDNA. Thus, MQC imbalance plays an important regulatory role in cell injury in the inflammatory state.

### 8.2. Effect of Inflammation on MQC

mtDNA is indispensable for energy metabolism and the regulation of cell death. ROS can damage mtDNA [168]. In the process of inflammation, ROS affect the mitochondrial structure, dynamics, and genomic stability, resulting in mtDNA mutation and mitochondrial dysfunction, and increasing the release of proinflammatory factors [169, 170]. Tumour necrosis factor- (TNF-) *α* affects the stability of mtDNA and mitochondrial function [171]. Damaged mitochondria release mtDNA into the cytoplasm, which causes inflammation, and mtDNA is released into the circulation after tissue inflammation. As an important factor of inflammation and the immune response, the increase in circulating mtDNA and the upregulation of TLR9 expression participate in experimental autoimmune myocarditis and TLR4 activation-mediated myocarditis [171].

Treatments with interleukin-6 (IL-6) and TNF-*α* lead to Drp-1 phosphorylation and mitochondrial translocation, resulting in abnormal mitochondrial fission in H9C2 cardiomyocytes [172]. Therefore, mitochondrial dysfunction is usually associated with GTPase Drp-1-mediated mitochondrial mitosis. Interestingly, inhibition of NF-*κ*B inflammatory signalling indirectly inhibits endothelial mitochondrial fission; thus, NF-*κ*B seems to be a signal of inflammatory mitochondrial fission in endothelial cells. In addition, salicylate seems to maintain the mitochondrion fission/fusion balance against TNF-*α* by inhibiting NF-*κ*B [172]. Thus, the NF-*κ*B cascade and mitochondrion fission pathway regulate MQC and endothelial cell inflammatory responses in an interdependent manner and effective MQC-regulatory drugs with anti-inflammatory and antioxidant actions are urgently needed to protect myocardial cells and endothelial cells.

### 8.3. Natural Antioxidants That Protect Myocardial and Endothelial Cells through MQC in the Inflammatory State

#### 8.3.1. Apigenin

Apigenin is a flavonoid antioxidant that exists mainly in plants of the families Verbenaceae and Selaginellaceae. It has antiviral and anti-inflammatory effects and is used for treating an HIV infection. Compared with other flavonoids, apigenin has low toxicity [173].

Inflammation is characterised by increased ROS production, dysfunction of mitochondrial energy metabolism, and abnormal immune function, which can lead to the occurrence of diseases. Apigenin can inhibit ROS production, restore the activity of mitochondrial complex I, stabilise mitochondrial function during inflammation, and reduce caspase-3 activity to suppress lipopolysaccharide- (LPS-) induced apoptosis in endothelial cells [174]. Apigenin protects mice against myocardial infarction. It regulates mitophagy via mir-103-1-5p and parkin, suppresses apoptosis in myocardial cells, and effectively reduces the myocardial infarction area [175].

#### 8.3.2. Ilexonin A

Ilexonin A is a pentacyclic triterpenoid isolated from the dried leaf of *Ilex latifolia* that has strong antioxidant and anti-inflammatory activities [172]. Ilexonin A activates Nrf2, increases the expression of proteosome 20S subunit beta 5 (PSMB5) and NO production, inhibits ROS production and the production of inflammatory cytokines induced by palmitate, inhibits Drp-1 expression and mitochondrial overfission, and protects endothelial cells. *Nrf2* knockout inhibits the induction of PSMB5 expression and eliminates the inhibition of ROS production and mitochondrial fission by ilexonin A. Thus, ilexonin A promotes PSMB5 expression in an Nrf2-dependent manner, thus inhibiting mitochondrial overfission to protect endothelial cell function in the inflammatory state [176].

#### 8.3.3. Allicin

Allicin is an organic sulphur-containing compound that mainly exists in the bulbs of onion and other Alliaceae plants. To date, two types of organic sulphur compounds have been isolated from garlic, which have shown antioxidative effects, plasma cholesterol-lowering, blood pressure-lowering, and platelet activity-inhibiting effects [177, 178]. As a vascular protective agent, allicin can protect endothelial cells by regulating MQC.

Allicin can significantly inhibit LPS-induced oxidative stress injury and inflammatory reactions in HUVECs. Allicin inhibits ROS and LDH overproduction, reduces lipid peroxidation, and improves antioxidant enzyme activities in the mitochondria. It restores the MMP, inhibits cytC release, and promotes ATP synthesis. It inhibits the expression of TNF-*α* and IL-8 and the adhesion of endothelial cells and increases the apoptosis of HUVECs induced by LPS. Allicin increases the expression of LXR-*α* and Nrf2 signalling in a dose-dependent manner. The effects of allicin on MQC regulation and endothelial cell protection are inhibited by siRNA-mediated knockdown of LXR-*α* [179], suggesting that the protective mechanism of allicin on endothelial cells is mediated by LXR-*α*.

*In vivo*, allicin suppresses the accumulation of interstitial collagen and type I/III collagens, ROS levels, protein carbonylation, and thiobarbituric acid-reactive substances, and increases GPX activity. In addition, allicin significantly increases the mRNA and protein levels of Nrf2, NQO-1, and *γ*-GCS, and prevents the occurrence of myocardial remodelling and the development of myocardial hypertrophy [180].

#### 8.3.4. Melatonin

Melatonin is an amine hormone mainly produced in the pineal gland of mammals and humans, and it also exists in many plants. Melatonin regulates the sleep-wake cycle and has strong antioxidant activity [181]. Melatonin has different effects on inflammation and mitochondrial function in endothelial cells. It inhibits abnormal NF-*κ*B activation, restores the MMP, and increases the expression of mitochondrial glutathione. It inhibits the expression of IL-6 and IL-8 and LPS-induced inflammatory injury in endothelial cells [182].

## 9. Lipid Toxicity

Lipid toxicity occurs when lipids accumulate in cells and tissues, and the cells and tissues cannot fully metabolise or store them. Lipid toxicity is closely related to diabetes, atherosclerosis, coronary heart disease, and heart failure [183]. In normal cells, fatty acid synthesis, transportation, and utilisation are in dynamic equilibrium. Free fatty acids (FFAs) can be produced by biochemical synthesis or hydrolysis of triglycerides and phospholipids. FFAs are important components of the cell membrane that can produce energy or signalling molecules through the process of *β*-oxidation, and participate in the mechanism of posttranslational protein modification and posttranscriptional protein regulation [184]. When the demand for FFAs increases, FFAs can enter cells via protein or nonprotein carrier pathways. Excess FFAs can be converted into triglycerides [185]. Adipocytes can store a large number of triglycerides, whereas nonadipocytes, such as myocardial cells and endothelial cells, can store only a limited amount. If triglycerides are overloaded, they will be dysfunctional, and apoptosis and necrosis will occur [186]. Lipid toxicity damages cardiomyocytes and endothelial cells mainly via oxidative stress.

### 9.1. Lipid Toxicity and OS

Lipid toxicity is closely related to oxidative stress. For example, *α*/*β*-polyunsaturated fatty aldehydes produced by oxidative stress participate in the modification of proteins, DNA, and RNA and important pathways of oxidative stress damage, including the unfolded protein response, endoplasmic reticulum stress, and DNA damage. In addition, although cellular and mitochondrial antioxidant systems can limit the production of some lipids, *α*/*β*-polyunsaturated fatty aldehydes cause serious mitochondrial energy metabolism dysfunction, eventually leading to MQC imbalance and apoptosis [187, 188].

Lipid peroxidation is the result of a hydroxyl radical attack of phospholipids and triglycerides. Mitochondria are considered the main source of H_2_O_2_. Superoxide anions are produced by complexes I and III and can be converted by SOD to H_2_O_2_, which can give rise to hydroxyl radicals. Triglycerides are the main target of hydroxyl radical-mediated attack and lipid-free radical formation. Lipid-free radicals are rapidly oxidised, resulting in lipid peroxidation of the acyl chain, which eventually leads to mitochondrial metabolic dysfunction and increases cell vulnerability [189, 190].

Lipid toxicity and high glucose often cooccur in diabetes mellitus complicated with CVD. FFAs can escape from adipocytes into the blood and accumulate heterotopically in nonadipocytes, causing lipid toxicity [191, 192]. Triglycerides can reduce the biological effects of insulin in muscle and liver, and cause insulin resistance. Triglyceride accumulation in pancreatic islets can lead to functional damage of *β* cells and dysfunction of insulin secretion stimulated by glucose. Thus, lipid toxicity may reduce glucose oxidation by increasing fatty acid oxidation, which leads to ROS overproduction and increased vulnerability of cardiomyocytes and endothelial cells [191]. Long-term mitochondrial or cellular metabolic disorders eventually lead to type 2 diabetes. Constitutive hyperglycaemia can also lead to increased FFA metabolism, and FFAs reduce endothelium-derived myocardial vasodilation, leading to a series of CVDs [193, 194].

### 9.2. Lipid Toxicity and MQC

The regulation of lipid metabolism is closely related to MQC in cardiomyocytes and endothelial cells [195]. In response to LPS, TNF-*α* and TFAM levels, nuclear accumulation of Nrf1, and PGC-1 expression are increased, mitophagy is stimulated, and the expression of withering markers is increased in adult rat cardiomyocytes [196]. Neonatal rat cardiomyocytes cultured in high-fat condition produce excessive ROS, including H_2_O_2_, causing abnormal MMP, resulting in myocardial cell damage. Hyperlipidaemia affects the MMP and ROS production of H9C2 cardiomyocytes [197].

Low-density lipoprotein (LDL), a lipoprotein particle that carries cholesterol into peripheral tissue cells, can be oxidised into oxidised low-density lipoprotein (ox-LDL). When ox-LDL is in excess, the cholesterol it carries accumulates on the arterial wall, which is the main cause of atherosclerosis [198]. Ox-LDL stimulates inflammatory activation and MQC imbalance in human artery endothelial cells [199]. It induces high mRNA expression of *TNF-α*, *IL-6*, and *IL-1β*, increases mtROS production, and destroys mtDNA and the MMP in these cells. In addition, it mediates TLR9/NF-*κ*B and NLRP3/caspase-1 activation, which leads to an increase in apoptosis in endothelial cells [200]. Therefore, it is necessary to find effective natural drugs to regulate oxidative stress and MQC.

### 9.3. Natural Antioxidants That Protect Myocardial and Endothelial Cells through MQC in Lipid Toxicity

#### 9.3.1. Chlorogenic Acid

Chlorogenic acid is a phenolic component in *Flos lonicerae* that has higher antioxidant capacity than caffeic acid. It has anti-inflammatory, hypolipidemic, and free radical-scavenging effects [201–203]. Chlorogenic acid increases SIRT1 deacetylase activity and AMPK/PGC-1 expression and alleviates oxidative stress injury and mitochondrial dysfunction induced by ox-LDL. Silencing of *SIRT1*, *AMPK*, and *PGC-1* reduces the protective effect of chlorogenic acid on endothelial cells, indicating that chlorogenic acid alleviates ox-LDL-induced mitochondrial dysfunction and improves the vulnerability of endothelial cells by activating SIRT1 and regulating PGC-1 signalling [204].

#### 9.3.2. Mangiferin

Mangiferin is a polyphenol compound with a xanthone skeleton that is mainly found in the seeds, leaves, flowers, and fruits of plants of the family Lacqueraceae [205]. Mangiferin has antioxidant, anti-inflammatory, and immunomodulatory effects [206, 207]. It has a certain protective effect on mitochondrial HK-II in vascular endothelial cells. HK-II also has an anticell death effect. In vascular endothelial cells, stimulation with the saturated fatty acid palmitate causes HK-II release from the mitochondria due to cell acidification. Mangiferin increases the activity of pyruvate dehydrogenase, reduces the accumulation of lactic acid, promotes Akt phosphorylation of HK-II, and prevents HK-II shedding from the mitochondria. Mangiferin also prevents mPTP opening, restores the MMP, and suppresses apoptosis, thus protecting vascular endothelial cells [208].

#### 9.3.3. Delphinidin-3-Glucoside

Delphinidin-3-glucoside inhibits LDL oxidation and platelet aggregation [209]. It reduces the ROS and superoxide anion production and mitochondrial dysfunction induced by ox-LDL, restores the MMP, and inhibits abnormal mPTP opening and the proliferation and apoptosis of primary HUVECs induced by ox-LDL. *In vitro* and *in vivo* studies have shown that delphinidin-3-glucoside can enter endothelial cells in a temperature-, concentration-, and time-dependent manner through sodium-dependent glucose transporter (SGLT1). It decreases apoptosis-related caspase-3 and Bax expression and increases Bcl-2 expression. siRNA-mediated knockdown of *SGLT1* or phloridzin treatment (an SGLT1 inhibitor) affects the protective action of delphinidin-3-glucoside on endothelial cells, indicating that delphinidin-3-glucoside regulates MQC through the SGLT1 pathway to protect endothelial cells [209].

#### 9.3.4. Melatonin

Melatonin protects endothelial cells from LPS-induced apoptosis, especially in the regulation of mitochondrial fission [210]. LPS-induced cytosolic Ca^2+^ overload can lead to the upregulation of Ca^2+^-dependent xanthine oxidase. High levels of xanthine oxidase expression and excessive ROS production can lead to Drp-1 phosphorylation at serine 616 and migration to the mitochondrial surface. Phosphorylated Drp-1 initiates mitochondrial fission, resulting in abnormal MMP, cytC leakage, and high caspase-9 expression. Melatonin can stimulate the AMPK pathway and SERCA2a expression, inhibit ROS overproduction and Ca^2+^ overload induced by xanthine oxidase, and regulate Drp-1 phosphorylation and mitochondrial fission/fusion balance, thus protecting HUVECs [210].

## 10. Future Research Directions

CVDs and microvascular diseases have high incidence and mortality rates. Although their pathological mechanisms are complex, they are closely related to the biological activities of cardiac myocytes and endothelial cells. New therapeutic and regulatory targets to improve the biological activities of myocardial cells and endothelial cells and restore their physiological functions under various stresses and in diseases are urgently needed. As shown in Figure 2, natural antioxidants can regulate MQC through different signalling pathways. As the main source of intracellular energy and an important participant in various signalling pathways, mitochondria play indispensable roles in cell survival and death and are important targets for the protection of myocardial cells and endothelial cells.

As shown in Figure 2, Figure 3, and Table 2, natural antioxidants can improve the vulnerability of myocardial and endothelial cells under stress, and provide a good reference for the treatment of CVDs and other vascular diseases. Although new natural antioxidants are being explored and experimental research on natural antioxidants for the treatment of various diseases by regulating MQC is ongoing, there remain many urgent problems to be solved.

### 10.1. Clinical Value of Natural Antioxidants

Compared with synthetic antioxidants, natural antioxidants are safer and more efficient. Their antioxidant and protective effects on cardiomyocytes and endothelial cells have been demonstrated in numerous *in vivo* and *in vitro* studies. In addition, natural antioxidants have many other pharmacological effects, such as cardiovascular protection, anti-inflammatory, antiviral, antitumour, and antiageing effects. They exhibit certain beneficial effects in improving mitochondrial function and energy metabolism, stabilising the MMP, regulating mitochondrial antioxidant enzyme activities, regulating mPTP, and protecting cardiomyocytes and endothelial cells. Accordingly, natural antioxidants are gaining increasing attention in research on CVDs, skin diseases, and ageing.

Currently, the large-scale application of natural antioxidants in clinical practice is still limited and most drugs are still in the experimental stage. In the future, efforts should be made to discover new raw material sources and monomers with antioxidant activity, and more genetic and clinical studies of natural antioxidants regulating MQC are needed to promote their clinical value. With the development of mitochondrial research, we may discover that MQC disorder is involved in more pathological mechanisms in human diseases. Although there are still controversies in clinical practice, the mutation and deletion of mitochondrial DNA may be an important reason for human ageing and disease development. In the future, how to use natural antioxidants in the clinic, to maintain the integrity of the mitochondrial genome, and to avoid inflammatory reaction caused by MQC disorder under oxidative stress will have profound guiding significance to reveal the aetiology of human diseases and improve clinical treatment.

### 10.2. Synergy of Natural Antioxidants

Numerous diseases present similar manifestations of mitochondrial dysfunction. Whether different pathologies share a common mechanism remains to be elucidated. Most natural antioxidants regulate MQC via similar mechanisms. It is currently unknown whether there are effective natural antioxidants that can simultaneously treat multiple diseases, with different targets. At present, various types of natural antioxidants are often used together in the clinic, and medicinal herbs contain various types of active ingredients, which makes it difficult to understand and utilise the synergistic effects of different active components on MQC regulation and simultaneously avoid antagonistic interactions. These are relevant issues that need to be addressed in future.

The combined effect of multiple antioxidants is often greater than that of a single drug at the same dose. Natural antioxidant components often have synergistic antioxidant effects, which are influenced by the drug concentration and reaction system. Therefore, future research should focus on synergistic effects between antioxidants, looking for efficient, low-toxicity compounds to meet clinical needs. At present, natural plants or herbs are usually used to extract antioxidants in the pharmaceutical industry. There are serious problems, such as lack of resources, backward extraction technology, and low content of active ingredients, which limit the popularisation and application of natural antioxidants. Therefore, in the future, we should explore more new sources of natural antioxidant raw materials, constantly improve the extraction of effective ingredients, the planting of natural antioxidant raw materials, and further clarify the synergistic effect of natural antioxidants, to improve their clinical value.

### 10.3. Targeting Experimental Research on Mitochondria

The effects of natural antioxidants on MQC have been studied mainly in animal and cell models, but few studies revealed the biological activity of natural antioxidants *in vitro* or by direct administration. It is difficult to judge whether natural antioxidants exert their effects by directly acting on mitochondria based only on animal and cell experiments. Therefore, the functions of natural drugs should be further investigated in isolated mitochondria to better understand their effect on MQC and their protective mechanism in myocardial cells.

Further, more in-depth studies should be conducted on the intake of natural antioxidants, dosing, bioavailability to the mitochondria, and tolerance of the intracellular environment. Interaction mechanisms among various stress conditions, such as high glucose, lipid toxicity, hypoxia, and ischaemia, remain to be elucidated. Causes and mechanisms of MQC disorders under stress conditions should be further explored to develop more effective natural antioxidants specifically targeting the MQC-regulatory effect and to provide more experimental evidence of and theoretical support for the mechanisms of natural antioxidants in protecting cardiomyocytes and endothelial cells.

### 10.4. Clinical Application of Mitochondrion-Targeted Therapy

The adverse consequences of oxidative stress and mitochondrial dysfunction mediated by various stresses seriously threaten the lives of patients with CVDs and bring great pressure to clinical treatment. Therefore, it is very important to analyse and summarise the targets and signalling pathways that regulate mitochondrial quality control and explore effective targeted therapies for MQC. In addition to natural antioxidants, mitochondrial transplantation, lifestyle intervention, and drug intervention can play effective roles in mitochondrial protection and restore or improve mitochondrial respiratory function and energy metabolism.

Mitochondrial transplantation is a new treatment for CVDs. It refers to the isolation of mitochondria from normal tissues and transportation of functional mitochondria to damaged tissues and organs to replace the damaged mitochondria and restore the normal mitochondria. This method can restore the normal structure and function of mitochondria in the clinic. In addition to natural antioxidants, some mitochondrion-targeted regulatory drugs, such as Mdivi1, P110, and Dynasore, can also reduce mitochondrial oxidative stress and improve mitochondrial function. Coenzyme Q10, which exists in the inner membrane of mitochondria, can also play an important role in ATP production and has certain antioxidant properties. Whether the combination of the above drugs and natural antioxidants can be effective needs more in-depth clinical research. In clinical practice, early effective MQC, reduction of mitochondrial dysfunction, and oxidative stress in CVDs are expected to become new targets in treatment strategy.

## 11. Conclusions

This review discussed the major effects of oxidative stress, hypoxia, I/R, inflammation, high glucose, and lipid toxicity on the MQC in cardiomyocytes and endothelial cells. These and other stress conditions induce excessive ROS production in these cell types, leading to MQC disorder and serious oxidative stress damage, which form an important mechanism in the development of CVDs and microvascular diseases. This review further explored the mechanism of 34 natural antioxidants in improving the vulnerability of cardiomyocytes and endothelial cells under stress by regulating MQC. Different types of natural antioxidants can maintain or restore the physiological function of mitochondria under stress by regulating MQC and improving cell viability and vulnerability. In conclusion, natural antioxidants have certain advantages in the regulation of MQC and the improvement of cardiomyocyte and endothelial cell activity and show promise as candidate drugs for clinical treatment of CVDs in future.

## Figures and Tables

**Figure 1:** Mechanism of oxidative stress-mediated by different stress conditions. Under stress conditions (small red rectangle), cells release free radicals (H_2_O_2_, NO, OH, and ONOO^−^), leading to the production of reactive oxygen species (ROS) and reactive nitrogen species (RNS). Excessive ROS and RNS production reduce the activity of antioxidant enzymes in the mitochondrial antioxidant system, causing ROS-mediated stress damage and the subsequent appearance of oxidative stress markers (red circles). H/R: hypoxia/reoxygenation; I/R: ischaemia/reperfusion; SOD: superoxide dismutase; GSH-Px: glutathione peroxidase; PRX: peroxiredoxin; CAT: catalase; MDA: malondialdehyde; 8-OHG: 8-hydroxyguanosine; 8-OHdG: 8-2′-hydroxydeoxyguanosine.

**Figure 2:** Mechanism of natural antioxidants that regulate MQC through different signalling pathways.

**Figure 3:** Mechanism of natural antioxidants in improving the vulnerability of cardiomyocytes/endothelial cells under stress by regulating mitochondrial quality control (MQC). (1) Different stress conditions can mediate severe oxidative stress damage and lead to MQC disorder, which further leads to increased vulnerability and apoptosis of cardiomyocytes and endothelial cells. This mechanism is reflected in many cardiovascular and microcirculation diseases. (2) Natural antioxidants can improve the quality and quantity of mitochondria by inhibiting the abnormal opening of the mitochondrial membrane permeability transition pore (mPTP), regulating the balance of mitochondrial lysis/fusion, regulating mitochondrial autophagy, and improving the function of the mitochondrial respiratory chain. It can also improve the vulnerability of myocardial cells and endothelial cells under stress, and provide a good reference for the treatment of cardiovascular diseases (CVDs) and other vascular diseases. H/R: hypoxia/reoxygenation; I/R: ischaemia/reperfusion; 8-OHdG: 8-2′-hydroxydeoxyguanosine.

**Table 1:** Effects of different stress conditions on MQC.

Stress condition	Impact on ROS	Effects on MQC of cardiomyocytes/endothelial cells	Natural antioxidants
Oxidative stress	Mitochondrial respiratory chain dysfunction leads to excessive ROS production	(1) Excessive mitochondrial fission (2) Mitochondrial Ca^2+^ homeostasis imbalance (3) Abnormal opening of mPTP (4) Mitochondrial respiratory dysfunction	(1) *P. notoginseng* saponins (2) Astragaloside IV (3) Cabbage extract (4) Mistletoe extracts (5) Tanshinone IIA (6) Ligustrazine (7) Resveratrol (8) Luteolin (9) Grape seed procyanidins
Hypoxia	Mitochondrial oxidative phosphorylation dysfunction leads to excessive ROS production	(1) Excessive mitochondrial fission (2) Mitochondrial Ca^2+^ homeostasis imbalance (3) Mitochondrial biosynthesis decreases (4) Loss of mitochondrial membrane potential	(1) Ginseng polysaccharide (2) Isoquercetin (3) Vitex flavonoids (4) Schisandrin/schisandrin B (5) Picroside (6) Anthocyanin
Ischaemia/reperfusion	Decoupling of the mitochondrial respiratory chain leading to excessive ROS production	(1) Mitochondrial Ca^2+^ homeostasis imbalance (2) Mitochondrial respiratory dysfunction (3) The level of mitochondrial ATP synthesis decreases	(1) *Panax quinquefolium* saponin (2) Ginsenoside RG5 (3) Lycopene (4) Cynomorium songaricum extract (5) Quercetin
High glucose	High levels of insulin interfere with NOX4 lead to excessive ROS production	(1) Excessive mitochondrial fission (2) Interference with the mitochondrial electron transport chain (3) Loss of mitochondrial membrane potential	(1) Naringin (2) Berberine (3) Cinnamaldehyde (4) Rosmarinic acid (5) Resveratrol (6) Pleurotus nebrodensis extract (7) Obtusin (8) Polydatin
Inflammation	Activated infiltrating immune cells and inflammatory resident cells lead to excessive ROS production	(1) mtDNA damage (2) Excessive mitochondrial fission	(1) Apigenin (2) Ilexonin A (3) Allicin (4) Melatonin
Lipid toxicity	Lipotoxicity increases the oxidation of fatty acids and leads to excessive ROS production	(1) Mitochondrial autophagy is inhibited (2) Loss of mitochondrial membrane potential (3) mtDNA damage	(1) Chlorogenic acid (2) Mangiferin (3) Anthocyanin (4) Melatonin

**Table 2:** Mechanisms of various natural antioxidants in protecting myocardial cells and endothelial cells under stress.

Natural antioxidant	Source	Chemical formula	Regulation mechanism of MQC	Stress condition	Targeted cells
Panax notoginseng saponins	*Panax notoginseng*	**—**	(1) Inhibits ROS overproduction (2) Upregulates forkhead box O3a and Mn-SOD expression (3) Upregulates expression of PGC-1 *α*, LC3-II, and Beclin-1	Oxidative stress	Cardiomyocytes
Astragaloside IV	*Astragalus propinquus*	C_41_H_68_O_14_	(1) Inhibits ROS overproduction (2) Inhibits LDH/creatine kinase MB isoenzyme/CytC release (3) Increases succinate dehydrogenase and ATPase activities (4) Induces phosphorylation of PI3K and Akt	Oxidative stress	Cardiomyocytes
Cabbage extract	*Daucus carota*	**—**	(1) Inhibits ROS overproduction (2) Enhances SOD-1, cat, and GPX activities (3) Inhibits MAPK (ERK1/2, JNK, and P-38) activation	Oxidative stress	Cardiomyocytes
Homoeriodictyol	*Citrus limon* etc.	C_16_H_14_O_6_	(1) Activates Nrf2 signalling (2) Restores MMP level (3) Inhibits CytC/apoptosis-inducing factor release (4) Inhibits caspase 3/9 overexpression (5) Increases the expression of Bcl-2 and Bcl-xL	Oxidative stress	HUVECs
Tanshinone IIA	*Salvia miltiorrhiza*	C_19_H_18_O_3_	(1) Increases mRNA levels of Mfn1 and OPA1 (2) Regulates the mitochondrial fission/fusion balance (3) Enhances GlO1 expression	Oxidative stress	Bovine retinal endothelial cells
Ligustrazine	*Ligusticum chuanxiong*	C_8_H_12_N_2_	(1) Inhibits CytC release (2) Restores the MMP level (3) Inhibits LDH	Oxidative stress	HUVECs
Resveratrol	*Polygonum cuspidatum*, *Vitis vinifera*, etc.	C_14_H_12_O_3_	(1) Inhibits ROS overproduction (2) Activates TyrRs-PARP1 and AMPK\PCG-*α*\Sirt3 signalling (3) Increases protein expression of Mfn1, Mfn2, and Opa1 (4) Regulates the mitochondrial fission/fusion balance (5) Increases IDH2, GSH-Px, and SOD2 activities	Oxidative stress	HUVECs
Luteolin	*Lonicera japonica* etc.	C_15_H_10_O_6_	(1) Restores MMP level (2) Regulates Ca^+^ homeostasis (3) Regulates p53 phosphorylation (4) Adjusts the Bcl-2/Bax ratio (5) Inhibits CytC release	Oxidative stress	Endothelial cells
Grape seed procyanidins	*Vitis vinifera*	C_30_H_12_O_6_	(1) Inhibits ROS overproduction (2) Restores the MMP level (3) Inhibits 8-OHdG expression (4) Enhances eNOS and VE-cadherin expression	Oxidative stress	HUVECs
Ginseng polysaccharide	*Panax ginseng* etc.	**—**	(1) Maintains the level of MMP (2) Inhibits CytC release (3) Improves mitochondrial respiratory function and ATP production (4) Activates risk signalling (5) Induces glucocorticoid and oestrogen receptor expression and enhances eNOS and iNOS expression	Hypoxia	Endothelial cells
Isoquercetin	*Hippophae rhamnoides*, *Crataegus pinnatifida*, etc.	C_21_H_20_O_12_	(1) Inhibits ROS overproduction (2) Improves the level of mitochondrial energy metabolism (3) Inhibits CytC release	Hypoxia	Cardiomyocytes
Vitex flavonoids	*Vitex quinata*	**—**	(1) Inhibits ROS overproduction (2) Inhibition of abnormal opening of MPTP (3) Inhibits CytC release and caspase-3 expression (4) Activates PI3K/Akt signalling (5) Adjusts the Bcl-2/Bax ratio	Hypoxia	Cardiomyocytes
Schisandrin/schisandrin B	*Schisandra chinensis*, *Schisandra sphenanthera*	C_24_H_32_O_6_/C_23_H_28_O_6_	(1) Inhibits abnormal opening of MPTP (2) Inhibits CytC release (3) Enhances GSH activity (4) Increases the cleavage of caspase-3 and poly ADP ribose polymerase	Hypoxia	Cardiomyocytes
Picroside	*Neopicrorhiza scrophulariiflora*	**—**	(1) Inhibits ROS overproduction (2) Inhibits abnormal opening of MPTP (3) Restores the MMP level (4) Inhibits CytC release (5) Downregulates caspase-3 expression	Hypoxia	Cardiomyocytes
Anthocyanins	Fruits, vegetables	**—**	(1) Restores the MMP level (2) Inhibits Bax transport to the nucleus (3) Inhibits the expression of caspases 3/9	Hypoxia	Endothelial cells
Panax quinquefolium saponin	*Panax quinquefolium*	**—**	(1) Inhibits abnormal MPTP opening (2) Regulates the mitochondrial Bcl-2/Bax ratio (3) Inhibits CytC release (4) Downregulates caspases 3/9 (5) Inhibits ROS overproduction	I\R	Cardiomyocytes
Ginsenoside Rg5	*Panax*	C_41_H_68_O_12_	(1) Inhibits fatty acid oxidation (2) Activates Akt signalling (3) Regulates Drp1 expression (4) Promotes HK-II mitochondrial binding	I/R	Cardiomyocytes
Lycopene	*Solanum lycopersicum*, *Punica granatum*, etc.	C_40_H_56_	(1) Inhibits 8-OHdG expression (2) Inhibits ROS overproduction (3) Recovers TFAM protein expression	I/R	Cardiomyocytes
Cynomorii extract	*Cynomorium songaricum*	**—**	(1) Increases mitochondrial ATP production (2) Enhances the redox cycle of glutathione (3) Inhibits expression of LDH and caspase-3	I/R	Cardiomyocytes
Quercetin	*Hippophae rhamnoides*, *Crataegus pinnatifida*, etc.	C_15_H_10_O_7_	(1) Restores the MMP level (2) Inhibits CytC release (3) Adjusts the Bcl-2/Bax ratio (4) Inhibits activation of caspases 3/9	I\R	HUVECs
Naringin	*Citrus grandis*	C_27_H_32_O_14_	(1) Inhibits p38 and p53 phosphorylation (2) Restores the MMP level (3) Inhibits CytC release (4) Adjusts theBcl-2/Bax ratio (5) Inhibits activation of caspases 3/8/9	High glucose	Cardiomyocytes
Berberine	*Coptis* etc.	C_20_H_18_NO_4_	(1) Regulates the mitochondrial fission/fusion balance (2) Activates AMPK signalling (3) Restores mitochondrial autophagy flux (4) Promotes mitochondrial biosynthesis	High glucose	Cardiomyocytes
Cinnamaldehyde	*Cinnamomum cassia*	C_9_H_8_O	(1) Inhibits ROS overproduction (2) Activates TRPA1/Nrf2 signalling (3) Enhances HO-1, GPx-1, and NQO-1 expression (4) Upregulates nitrotyrosine, P22, and P47 expression	High glucose	Cardiomyocytes
Rosmarinic acid	*Rosmarinus*	C_18_H_16_O_8_	(1) Inhibits ROS overproduction (2) Inhibits abnormal mPTP opening (3) Inhibits CytC release and caspase-3 activation (4) Increases STAT3 phosphorylation	High glucose	Cardiomyocytes
Resveratrol	*Polygonum cuspidatum*, *Vitis vinifera*, etc.	C_14_H_12_O_3_	(1) Inhibits ROS overproduction (2) Activates SIRT1 signalling (3) Upregulates Mn-SOD expression and GSH activity	High glucose	Human coronary artery endothelial cells
Obtusifolin	*Cassia tora*	C_16_H_12_O_5_	(1) Inhibits ROS overproduction (2) Inhibits electronic transport chain complex I activity (3) Regulates SOD and CAT activities	High glucose	HUVECs
Polydatin	*Polygonum cuspidatum*	C_20_H_22_O_8_	(1) Inhibits ROS overproduction (2) Restores the MMP level and morphological changes of mitochondria (3) Increases Akt phosphorylation	High glucose	Endothelial cells
Apigenin	*Apium graveolens*	C_15_H_10_O_5_	(1) Inhibits ROS overproduction (2) Recovers mitochondrial complex I activity (3) Decreases caspase-3 expression (4) Adjusts miR-103-1-5p and parkin (5) Regulates mitochondrial autophagy	Inflammation	Cardiomyocytes
Ilexonin A	*Ilex pubescens*	C_36_H_56_O_11_	(1) Activates Nrf2 signalling (2) Enhances PSMB5 expression (3) Inhibits ROS overproduction (4) Inhibits abnormal mitochondrial fission	Inflammation	Endothelial cells
Allicin	*Allium sativum*	C_6_H_10_OS_2_	(1) Inhibits ROS/LDH/thiobarbituric acid-reactive substance overproduction (2) Restores the MMP level (3) Inhibits CytC release (4) Inhibits TNF-*α* and IL-8 expression (5) Activates LXR-*α* and Nrf2 signalling	Inflammation	Endothelial cells
Melatonin	**—**	C_13_H_16_N_2_O_2_	(1) Inhibits abnormal NF-*κ*B activation (2) Restores the MMP level (3) Increases glutathione expression in mitochondria (4) Inhibits IL-6 and IL-8 expression	Inflammation	Endothelial cells
Chlorogenic acid	*Lonicera japonica* etc.	C_16_H_18_O_9_	(1) Increases SIRT1/AMPK/PGC-1 expression (2) Inhibits ROS overproduction (3) Decreases caspase-3 expression (4) Adjusts the Bcl-2/Bax ratio	Lipid toxicity	Endothelial cells
Mangiferin	*Mangifera indica*	C_19_H_18_O_11_	(1) Increases pyruvate dehydrogenase activity (2) Promotes translocation of Akt to HK-II (3) Inhibits abnormal mPTP opening (4) Restores the MMP level	Lipid toxicity	Endothelial cells
Anthocyanin	Fruits, vegetables	**—**	(1) Restores the MMP level (2) Inhibits abnormal mPTP opening (3) Inhibits CytC release (4) Decreases caspase-3 and Bax expression	Lipid toxicity	HUVECs
Melatonin			(1) Activates AMPK/SERCA2a signalling (2) Inhibits ROS overproduction and Ca^+^ overload (3) Regulates Drp1 phosphorylation (4) Regulates the mitochondrial fission/fusion balance	Lipid toxicity	HUVECs

## Data Availability

The data used to support the findings of this study are included within the article.
